The article "Desensitization of ABA-Signaling: The Swing From Activation to Degradation" was published in 2020. Journal: Front Plant Sci.

# Desensitization of ABA-Signaling: The Swing From Activation to Degradation

**DOI:** 10.3389/fpls.2020.00379

**Published:** 2020-04-22

**Authors:** Akhtar Ali, Jose M. Pardo, Dae-Jin Yun

**Affiliations:** ^1^Department of Biomedical Science and Engineering, Konkuk University, Seoul, South Korea; ^2^Instituto de Bioquímica Vegetal y Fotosíntesis, cicCartuja, CSIC-Universidad de Sevilla, Seville, Spain

**Keywords:** ABA-signaling, ABA core proteins, protein degradation and stability, HOS15, OST1

## Abstract

Abscisic acid (ABA) is a key plant stress-signaling hormone that accumulates upon osmotic stresses such as drought and high salinity. Several proteins have been identified that constitute the ABA-signaling pathway. Among them ABA receptors (PYR/PYL/RCAR), co-receptor PP2Cs (protein phosphatases), SnRK2 kinases (SNF1-related protein kinases) and ABI5/ABFs (transcription factors) are the major components. Upon ABA signal, PYR/PYL receptors interact with and recruit PP2Cs, releasing SnRK2s kinases from sequestration with PP2Cs. This allows SnKR2s to promote the activation of downstream transcription factors of ABA pathway. However, apart from activation, ubiquitination and degradation of core proteins in the ABA pathway by the ubiquitin proteasome system is less explored. In this review we will focus on the recent findings about feedback regulation of ABA signaling core proteins through degradation, which is emerging as a critical step that modulates and eventually ceases the signal relay. Additionally, we also discuss the importance of the recently identified effector protein HOS15, which negatively regulate ABA-signaling through degradation of OST1.

## Introduction

Being sessile by nature, plants have evolved the ability to alter their physiology and development to adapt to the environmental challenges (Bohnert et al., 1995). Unfavorable conditions, such as high salinity, cold or drought stress, are important challenges to agriculture as they reduce the yield potential of crop plants. Phytohormones play a pivotal role in environmental adaptation by inducing many biochemical and physiological changes to respond to biotic and abiotic stresses (Cao et al., 2011; Seo et al., 2014; Pozo et al., 2015). Among them, abscisic acid (ABA) is an important regulator of plant growth and development that also plays a crucial role in both biotic and abiotic stress responses (Lee et al., 2006; Adie et al., 2007; Mang et al., 2012; Finkelstein, 2013). ABA regulates multiple physiological processes such as seed maturation, embryo morphogenesis, and stomatal movement to rescue plants under water deficit condition (Yoshida et al., 2002; Finkelstein, 2013; Murata et al., 2015). The phenotypes of the ABA-defective mutants (both in synthesis and/or signaling), which included loss of seed dormancy and early seedling growth and loss of stomatal movement, supported the importance of ABA in developmental and physiological responses (Koornneef et al., 1982; Lee et al., 2006; Finkelstein, 2013).

The article "Desensitization of ABA-Signaling: The Swing From Activation to Degradation" was published in 2020. Journal: Front Plant Sci.

In response to environmental stresses ABA levels rise and set in motion the adaptive stress responses (Zabadal, 1974; Lee et al., 2006; Hua et al., 2012). The perception of ABA is achieved by a family of ABA receptors named Pyrabactin Resistance (PYR), or Regulatory Component of ABA Receptor (RCAR) (Ma et al., 2009; Park et al., 2009). In the presence of ABA, the ABA receptors PYR/PYL(PYR-Like)/RCAR function at the apex of a negative regulatory pathway to directly bind to and inactivate type 2C Ser/Thr protein phosphatases (PP2Cs) (Geiger et al., 2009; Ma et al., 2009; Park et al., 2009; Rodrigues et al., 2013). This allows the activation of SnRK2 kinases (Snf1-related protein kinase class 2), which subsequently phosphorylate ABI5/ABFs transcription factors (ABA-Insensitive5/ABA-responsive element binding factors) (Fujii et al., 2009). However, negative effectors that modulate the intensity of the response, and which will eventually cancel the signaling cascade, must also come into action to counteract this positive signal relay and prevent a run-away process. Finely controlled protein stability is emerging as a novel critical regulatory layer accounting for signal termination, and also for desensitization upon repeated or sustained stimuli. Here, we summarize recent insights into controlled protein degradation of signaling effectors of the ABA pathway, with an emphasis on the newly discovered player HOS15, a component of the protein ubiquitination machinery that tags SnRK2.6/OST1 and histone deacetylase 2C (HD2C) for degradation, thereby modulating ABA signaling, chromatin status and gene expression in response to dehydration and cold stresses in Arabidopsis (Park et al., 2018; Ali et al., 2019).

## Ubiquitin Proteasome System (UPS)

Protein degradation by the Ubiquitin Proteasome System (UPS) is an important posttranslational regulatory step that controls protein stability and turnover. Protein ubiquitination combines activities of three enzymes, E1 (ubiquitin-activation), E2 (ubiquitin-conjugation), and E3 (ubiquitin ligase) (Pintard et al., 2004; Hotton and Callis, 2008). Target specificity is conferred by E3 ligases, and hence the Arabidopsis genome contains over 1400 genes encoding E3 ligases, which are classified into two groups (Vierstra, 2009). One group acts as a single subunit, which consists of RING-type (Really Interesting New Gene) E3 enzymes. The other group, which functions as a multi subunit complex, includes SCF (Skp1-Cullin-F-box) and APC (Anaphase Promoting Complex) (Vierstra, 2009). In the recent past, a number of RING-type E3 ligases were identified in Arabidopsis that were shown to be involved in various cellular processes, such as hormones signaling (auxin and ABA), seed germination and early seedling development and adaptive pathway to water limitation (Xie et al., 2002; Zhang et al., 2005, 2008; Stone et al., 2006; Bu et al., 2009; Huang et al., 2010). Among them, CULLIN4 (CUL4) has been described in greater detail due to its major role in different biological pathways. CUL4 interacts with DDB1 (DAMAGED DNA BINDING PROTEIN1) and a WD40-repeat protein as its substrate receptor (He et al., 2006; Hotton and Callis, 2008; Hua and Vierstra, 2011; Seo et al., 2014). The WD40-repeat (also known as the ß-transducin repeat) is a structural motif that folds as a solenoid-like structure called the WD40 domain. WD40-repeat proteins function as to facilitate multi-protein complex assemblies, where they serve as the scaffold for protein-protein interactions, including those of E3 ubiquitin ligases with target proteins. The Arabidopsis protein HOS15 (HIGH OSMOTIC STRESS GENE EXPRESSION 15) is a substrate receptor for the CULLIN4 (CUL4)-based ubiquitin E3 ligase that plays a negative role on ABA signaling and plant acclimation to cold (Lee et al., 2008; Zhu et al., 2008; Park et al., 2018). In the cold-stress response, HOS15 functions to mediate the cold-induced degradation of histone deacetylase 2C (HD2C) in the promoters of the COLD-RESPONSIVE (*COR*) genes. Enhanced histone acetylation switches the chromatin from an “open” status that facilitates recruitment of CBF (C-REPEAT BINDING FACTOR) transcription factors to the *COR* genes (Park et al., 2018). We have recently shown that HOS15 also plays a substantial role in regulating the signaling flux in response to ABA by controlling the protein stability and abundance of intermediaries in the pathway (Ali et al., 2019).

The article "Desensitization of ABA-Signaling: The Swing From Activation to Degradation" was published in 2020. Journal: Front Plant Sci.

PYR/PYL/RCAR (ABA receptors), PP2Cs (phosphatases), SnRKs (SNF1-related protein kinases) and ABI5/ABFs (transcription factors) are major components of forward ABA-signaling (Fujii and Zhu, 2009; Park et al., 2009). Ten SnRK2 members (SnRK2.1 to SnRK2.10) have been identified in Arabidopsis (Hrabak et al., 2003), with three of them (SnRK2.2/2.3/2.6) being activated by ABA (Fujita et al., 2009). Among the three, SnRK2.6/OST1 specifically regulates water loss through stomata (Yoshida et al., 2002; Hua et al., 2012). Evidence is emerging that ubiquitination and degradation of these ABA-signaling components is of upmost importance to fully understand that how this signaling pathway is modulated and eventually ceased (Table 1).

**TABLE 1:** List of E3 ligases (and other proteins/linkers) which regulate protein level of ABA signaling core components.

**E3 ligases/Linkers**	**Target protein**	**Published by**
AFP1	ABI5	Lopez-Molina et al., 2003
DWA1/DWA2	ABI5	Lee et al., 2010
KEG	ABI5/ABF1/3	Liu and Stone, 2013; Chen et al., 2013
ABD1	ABI5	Seo et al., 2014
RSL1	PYL4/PYR1	Bueso et al., 2014
DDA1	PYL4/8/9	Irigoyen et al., 2014
ALIX	PYL4/5/8/L9	García-León et al., 2019
RIFP1	RCAR3	Li et al., 2016
REA1	PYL9	Li et al., 2018
PUB22/PUB23	PYL9	Zhao et al., 2017
FYVE1	PYL4	Belda-Palazon et al., 2016
VPS23A	PYR1/PYL4	Yu et al., 2016
PUB12/PUB13	ABI1	Kong et al., 2015
RGLG1/RGLG5	PP2CA	Wu et al., 2016
PIR1/PIR2	PP2CA	Baek et al., 2019
BPM3/BPM5	ABI1/PP2CA/HAB1	Julian et al., 2019
PP2B11	SnRK2.3	Cheng et al., 2017
HOS15	OST1	Ali et al., 2019

## ABA Receptors (PYR1/PYL/RCAR)

Several reports in the recent past have shown that ABA receptors are degraded by a number of E3 ligases in an ABA-dependent manner (Table 1). Sorting and vacuolar degradation of ABA receptors are mediated by components of the ESCRT machinery (Endosomal Sorting Complex Required for Transport), i.e., FYVE1 and VPS23A (Belda-Palazon et al., 2016; Yu et al., 2016). ALIX (ALG-2 INTERACTING PROTEIN-X), another ESCRT protein, directly interact with ABA-receptors (PYL4/5/8/9) in late endosomes and promote their degradation (García-León et al., 2019). Furthermore, genetic interference with ALIX function leads to altered endosomal localization and increased accumulation of ABA receptors, indicating that to perform normal function, inhibition of ABA-receptor’s over-accumulation needs to be carried out (García-León et al., 2019). Degradation of RCAR1/PYL9 mediated by PUB22 and PUB23 (U-box E3 ligases) has recently been shown (Zhao et al., 2017). Additionally, RAE1, a WD40 repeat protein, and RIFP1, an adaptor subunit of the SCF ubiquitin ligase complex, promote the degradation of RCAR1 and RCAR3, respectively (Li et al., 2016, 2018). Based on these reports one can easily assume that regardless of their positive role, controlled turnover of ABA-receptors at protein level is a critical step that fine tunes ABA-signaling pathway. The reason why degradation of the ABA receptors and of other signaling intermediaries (Table 1) is redundantly achieved by several types of E3 ligases is presently unknown. Likely, seemingly redundant ways leading to protein degradation reflect the diversity of developmental and physiological processes in which the target proteins participate or their diverse subcellular locations (see below).

The article "Desensitization of ABA-Signaling: The Swing From Activation to Degradation" was published in 2020. Journal: Front Plant Sci.

## Protein Phosphatases (ABI/HAI/HAB)

Next to ABA receptors, protein phosphatases (PP2Cs), acting as co-receptors of ABA, have emerged as important regulators of ABA-signaling. Primarily, PP2Cs function as inhibitors of ABA-signaling pathway through inactivation of SnRK2 kinases (Brandt et al., 2012). Members of protein phosphatases PP2Cs that include ABI1/2, HAB1/2, HAI1/2/3, and AHG1/3 sequester SnKR2 kinases, inhibiting their kinase activity and thus functions as negative regulators of ABA-signaling. To release from sequestration by PP2Cs, SnRK2 kinases require ABA binding to PYR1/PYL/RCAR receptors (Fujii et al., 2009). Furthermore, increased or decreased phosphatase activities of these PP2Cs result in altered ABA responses that are SnRK2-dependent. For instance, knock out mutants of PP2Cs such as *abi1-2* display enhanced ABA signaling, whereas dominant-negative mutations of the same PP2C (*abi1-1*), lead to suppression of ABA-signaling in a SnRK2s-dependent manner (Umezawa et al., 2009). PP2Cs are also regulated through proteasomal degradation. Degradation of ABI1, a well-known protein phosphatase in the ABA-signaling, has been reported (Kong et al., 2015). PUB12/PUB13 (U-box E3 ligases) interact with ABI1 and are able to ubiquitinate ABI1 in the presence of ABA. The ubiquitinated ABI1 is degraded by the 26S proteasome (Kong et al., 2015). Beside ABI1, the degradation of PP2CA, another phosphatase that negatively regulate SnRK2s activity, was recently reported, which is mediated by the RING finger E3 ligases RGLG1/RGLG5 and PIR1/PIR2 (Wu et al., 2016; Baek et al., 2019). In all these cases, E3 ligases positively modulate ABA signaling by targeting the phosphatases for degradation, thereby amplifying the signal flux.

As with the ABA receptors, more than one E3 ligase modifies a single substrate depending on the physiological context (Hare et al., 2003; Liu and Stone, 2010; Cheng et al., 2012; Seo et al., 2014). For instance, PP2CA protein stability is modulated by both RGLG1/5 and PIR1/2 (Wu et al., 2016; Baek et al., 2019). However, compared with RGLG1/5, PIR1 and PIR2 can strongly interact with PP2CA in the absence or the presence of low ABA, suggesting that PIR1 and PIR2 may regulate PP2CA protein stability under non-stress conditions (Wu et al., 2016; Baek et al., 2019).

## Snf1-Related Kinases2 (SnRk2s)

Although Snf1-Related Kinases (SnRK2s) kinases are major components that regulate ABA-signaling pathway, little is known about the feedback regulation of SnRK2s in post-ABA condition to terminate the signal. Overall, de-activation of SnRK2s at protein level, has been less studied and only few reports are available to date (Table 1). Upon ABA signal, activated SnRK2s phosphorylate and activate target proteins including ABF transcription factors (Fujita et al., 2009). Interestingly, the activated ABFs bind to the promoters of *ABI1* and *ABI2* genes and promote their transcription, thereby controlling SnRK2s activity through a negative feedback regulation loop (Wang et al., 2018). Besides dephosphorylation by PP2Cs, AtPP2-B11, a component of the SCF ubiquitin E3 ligase complex, has been shown to promote the ABA-dependent ubiquitination and degradation of SnRK2.3 (Cheng et al., 2017). More recently, we have also shown that the degradation of SnRK2 kinases is really important for the controlled turnover of ABA signal relay. Using yeast two hybrid screen, we identified that HOS15 interacts specifically with OST1, SnRK2.3 and ABI1/2 (and very weakly with HAI1). Further analysis showed that HOS15 specifically interacts with OST1 in an ABA-dependent manner and promotes its degradation (Ali et al., 2019). OST1 level was highly accumulated in *hos15-2* plants, which leads to significant tolerance to drought stress (Ali et al., 2019).

The article "Desensitization of ABA-Signaling: The Swing From Activation to Degradation" was published in 2020. Journal: Front Plant Sci.

## Involvement of HOS15 in ABA-Signaling Pathway

HOS15, a substrate receptor in the CUL4-DDB1 E3 ligase machinery, negatively regulate ABA-signaling and drought stress by interference with OST1 stability (Ali et al., 2019). HOS15 was found to interact with ABI1, ABI2, and OST1; however, only HOS15 and OST1 interaction was diminished by ABA (Ali et al., 2019). OST1 level was remarkably stable and accumulated in *hos15-2* compared to wild type (Columbia-0) plants, demonstrating that HOS15 negatively regulates OST1 stability, presumably leading to termination of ABA signaling (Ali et al., 2019). Loss-of-function *hos15-2* mutant plants are hyper-sensitive to ABA during germination and extremely tolerant to drought stress, indicating the importance of HOS15 as a negative regulator (Ali et al., 2019). Moreover, ABA- and dehydration stress-responsive genes were highly induced in *hos15-2* plants under dehydration stress (Ali et al., 2019). Since HOS15 plays a major role in ABA-signaling network, we were interested to place HOS15 in the current model of ABA-signaling pathway. Under normal condition ABI1/2 inhibits OST1 activity by dephosphorylating it (Yoshida et al., 2006; Park et al., 2009). In the presence of ABA, PYR1 inhibits ABI1, releasing OST1 that auto-phosphorylates itself and then *trans-*phosphorylate the target TFs (Antoni et al., 2012). Furthermore, ABA also impairs HOS15 and OST1 interaction (Ali et al., 2019), indicating that in the presence of ABA, inhibitory components are kept stay-away from OST1 (and other SnRK2s) that phosphorylate and activates ABA responsive components. By contrast, ABA has no clear effect on HOS15 interaction with ABI1 and ABI2 (Ali et al., 2019), demonstrating that once the ABA pathway is activated, OST1 is released from the HOS15-ABI1/2 complex. However, when ABA-pathway is about to turn-off, ABI1/2 promotes HOS15 and OST1 interaction, which leads to OST1 degradation (Figure 1). Importantly, we found that under sustained ABA stimulus, activated OST1 promoted *de novo* synthesis and accumulation of ABI1/2, which in turn dephosphorylated and promoted the degradation of OST1 (Figure 1). Accordingly, de-phosphorylated OST1 was the preferred substrate for HOS15 (Ali et al., 2019). Together, these functional and physical interactions depict the activity of a biological rheostat that through quantitative and mutual regulation of both positive and negative effectors achieves the adaptive modulation of signal amplitude and duration. In summary, HOS15 plays a crucial role in regulating ABA-signaling by degradation of OST1 and thus keeping a balance between active and inactive state.

The article "Desensitization of ABA-Signaling: The Swing From Activation to Degradation" was published in 2020. Journal: Front Plant Sci.

**FIGURE 1:** HOS15 negatively regulates ABA signaling through OST1 degradation. **Resting state:** Under normal condition ABI1/2 and HOS15 interact with OST1. ABI1/2 inhibits OST1 activity by de-phosphorylation and HOS15 degrades OST1 to keep it in a resting state. **Activation phase:** In response to ABA, PYR1 binds to ABA thus interacting with and inhibiting ABI1, releasing OST1 from sequestration with ABI1/2. HOS15 and OST1 interaction is diminished by ABA, which leads to OST1 activation. OST1 is first auto-phosphorylated and then *trans-*phosphorylates target TFs. **De-activation:** After removal of ABA from the system (4 h later), ABI1/2 again interacts (reverse reaction) with and dephosphorylates OST1, recruiting HOS15 to OST1 for degradation. Note that HOS15 also degrades OST1 within hours of sustained ABA treatment by a mechanism that involves ABI1/2 upregulation and dephosphorylation of OST1, leading to ABA de-sensitization (Ali et al., 2019).

## ABFs/ABI5

Activation of ABFs/ABI5 transcription factors (TFs) by SnRK2s completes the signal relay and links ABA signaling with ABA-dependent gene activation. Like their activation by phosphorylation, degradation of ABFs/ABI5 TFs by 26S proteasome has also been studied in detail (Table 1 and Figure 2). The first evidence regarding degradation of ABFs/ABI5 TFs was the identification of ABI FIVE BINDING PROTEIN1 (AFP1), a member of a small plant-specific protein family. AFP1 directly binds to ABI5 and facilitates ubiquitin-mediated proteolysis of ABI5 (Lopez-Molina et al., 2003). More recently, a number of E3 ligases and WD40-repeat proteins have been identified as negative regulators of both ABFs and ABI5 (Table 1). KEG (KEEP ON GOING), a RING-ANK E3 ligase, is required for the regulation of ABI5/ABF1/ABF3 abundance (Chen et al., 2013; Liu and Stone, 2013). *In vivo* studies have shown that in the absence of ABA, KEG ubiquitinate ABF1/ABF3/ABI5, and promotes proteasomal degradation of them (Liu and Stone, 2013). In addition, DWA1 and DWA2 (DWD hypersensitive to ABA1/2) are substrate receptors for the DDBI CULLIN4-based E3 ligases that directly interact with ABI5 and mediate the degradation of ABI5 by ubiquitination (Lee et al., 2010). More recently, Seo et al. (2014) found that ABD1, a WD40-repeat protein, directly interacts with and degrades ABI5. These reports indicate that activation and degradation of ABA-signaling components are critical processes that regulate ABA signaling pathway in a very fine way and that both processes are important alike.

The article "Desensitization of ABA-Signaling: The Swing From Activation to Degradation" was published in 2020. Journal: Front Plant Sci.

**FIGURE 2:** ABA signaling core proteins and their correspondent E3 ligases. In response to ABA, PYR/PYLs bind ABA, which promotes their interaction with PP2Cs and the release of SnRK2s from sequestration by PP2Cs. Activated SnRK2 kinases phosphorylate target transcription factors that induce the expression of ABA responsive genes. On the right side, E3 ligases are shown which have been shown to promote the degradation of ABA signaling core proteins.

## Conclusion

The plant hormone abscisic acid (ABA) controls a number of developmental processes including seed maturation, germination, embryogenesis, plant growth and development, and senescence (Zabadal, 1974; Lee et al., 2006; Finkelstein, 2013; Murata et al., 2015; Zhao et al., 2016). Several proteins were identified that work together to regulate ABA signaling including ABA-receptors and co-receptors, kinases and TFs (Fujii et al., 2009; Fujita et al., 2009; Park et al., 2009; Brandt et al., 2012). Activation and de-activation (degradation) of these proteins got huge attention in the recent past (Figure 2); however, compared to activation, little is known about degradation of these proteins. This review sheds light on the recent studies that focused on the degradation of ABA-signaling core components. Further investigations on how different E3 ligases are activated to degrade ABA core proteins, are the future goals.

## Author Contributions

D-JY and JP designed work. AA, JP, and D-JY collected information from literature and wrote the manuscript. All authors reviewed and approved the final manuscript.

## Conflict of Interest

The authors declare that the research was conducted in the absence of any commercial or financial relationships that could be construed as a potential conflict of interest.
